The article "Effect of Calcar Screw in Locking Compression Plate System for Osteoporotic Proximal Humerus Fracture: A Finite Element Analysis Study" was published in 2022. Journal: Biomed Res Int.

# Effect of Calcar Screw in Locking Compression Plate System for Osteoporotic Proximal Humerus Fracture: A Finite Element Analysis Study

**DOI:** 10.1155/2022/1268774

**Published:** 2022-09-15

**Authors:** Jung-Soo Lee, Jong Hoon Kim, Kwang Gi Kim, Yong-Cheol Yoon

**Affiliations:** ^1^Department of Health Sciences and Technology, Gachon Advanced Institute for Health Sciences and Technology (GAIHST), Gachon University, Incheon 21999, Republic of Korea; ^2^Department of Biomedical Engineering, College of Medicine, Gachon University, Incheon 21565, Republic of Korea; ^3^Medical Devices R&D Center, Gachon University Gil Medical Center, Incheon 21565, Republic of Korea; ^4^Orthopedic Trauma Division, Trauma Center, Gachon University Gil Medical Center, Incheon 21565, Republic of Korea

## Abstract

This study proposes a finite element analysis (FEA) model for complex fractures at the osteoporotic proximal humerus and investigates the relevance of using a calcar screw in surgical treatments using this model. Two types of three-dimensional (3D) fracture models of patients with osteoporotic humerus were constructed reflecting the mechanical properties of the osteoporotic humerus, such as the Young's modulus and Poisson's ratio, and two load conditions mimicking the clinical environment were applied for simulation. Using the 3D models and the conditions, the FEA software calculated the concentration and distribution of stresses developing in the humerus, locking compression plate (LCP), and screws. Then, we evaluated and predicted the fixed state of a LCP system depending on whether the maximum stress value exceeded tensile strength. When axial force was applied, insertion of the calcar screw led to significant reduction of stress applied on screws in the fracture model having a medial gap by approximately 61%, from 913.20 MPa to 351.84 MPa. Based on the results, it was clearly confirmed that using of calcar screws improved the stability of a three-part fractures and simultaneously reinforced medial support.

## 1. Introduction

Fractures of the proximal humerus account for approximately 5% of all fractures, and when osteoporotic patients fall, fracture is more likely to occur [1]. The majority of the elderly having low bone density are particularly vulnerable to such accidents. Considering the accelerated aging of the population in many countries, developing treatments that guarantee satisfactory recovery of such patients is urgent. Surgery is considered the only reliable approach for approximately 20% of patients with severe fractures [2], but the existing surgical treatments may be inadequate due to complications varying with the characteristics of the fractures [3].

Indeed, a comminuted fracture, i.e., fracture into multiple pieces, occurs frequently in osteoporotic patients and makes restoration of the bone to its original state difficult. Screw fixation in case of a comminuted fracture or for osteoporotic patients significantly increases the rate of complications such as reduction loss, fixation failure, malunion and nonunion of fracture, impingement syndrome, or avascular necrosis of the humeral head [4]. Considering the most suitable treatment for compound fractures, extramedullary plate fixation, consisting of a metal plate and screws, has long been used as a safe surgical method for fracture fixation [5]. Moreover, introduction of the locking compression plate (LCP) paved way for more stable and durable fixation of an osteoporotic proximal humerus fracture. The LCP technique permits merging of the locking screw system with the conventional plating technique through use of multiple small-angled blade plates for more durable binding and remarkable reduction in fixation failure. Therefore, bone fixation surgery using an LCP is considered the standard treatment owing to its accurate anatomical reduction and strong initial fixation of diaphysis fractures [6–8].

To broaden its application to diverse clinical cases and prove its effectiveness through quantitative analysis, this surgical procedure has been vigorously investigated [9–11] with a focus on the design of the LCP and on the appropriate number of screws for preventing bone loss [12–16]. The existing literature shows that placement of a calcar screw in the lower part of the proximal humerus can help achieve safe and stable fixation; using calcar screws particularly make sense in case of a fracture in which there is unstable medial support of the proximal humerus caused by the varus of humeral head. The calcar screw plays a key role for supporting and tightly fixing the fracture area having the defect of the posteroinferior calcar [17–20].

Many clinical studies and biomechanical experiments have attempted to demonstrate the importance of the medial support in humerus fractures [3, 8, 21]; however, there is a lack of quantitative studies such as FEA on alternatives for medial cortical support or studies analyzing the utility of a calcar screw as an effective reinforcement providing medial support to the proximal humerus in terms of comminuted fractures in osteoporotic elderly patients.

To address this issue, we used finite elements analysis (FEA) based on the idea that any complicated object can be virtually reconstructed with small and finite number of fundamental building blocks. Thus, its mechanical performance can be quantitatively and accurately analyzed, given that the mechanical properties and boundary conditions are fully defined.

We aimed to evaluate the effect of calcar screws through FEA simulations and provide quantitative evidence to aid decision-making during the clinical application of calcar screws based on the three-dimensional (3D) bone models of an elderly patient prepared according to the aforementioned considerations.

## 2. Material and Methods

### 2.1. Data Preparation

Computed tomography images of 50 patients with osteoporosis, aged > 60 years, were acquired from the Picture Archiving and Communication System (PACS) of the Department of Radiology, Gil Medical Center, Gachon University. Of the patients, there exist cases related to three-part or over three-part fractures, which normally require surgical treatments using LCP. The three-part fracture is characterized as being typically broken down to the surgical neck, greater tubercle, and shaft. In addition, the fractures frequently contain medial gaps in the surgical neck of the humerus as displayed in Figure 1(d). Of the different types of three-part fractures, we aimed to examine two kinds of osteoporotic fracture models, those with and without a medial gap in the surgical neck, as it could be a key feature to verify the effectiveness of LCP systems. In fact, these fracture modes have been subject to the majority of FEA studies examining the fixation state of LCP systems. Prior to the construction of an FE model, to ensure the reliability of the simulation, we chose the data amenable to FE modeling from four patients that were distinctly split into four main components of proximal humerus.

The fracture model for FEA simulation was created via preprocessing of raw data that is outlined in the following description.

First, the data of the humerus was divided into four regions, i.e., cortical bone, trabecular bone, articular cartilage, and subchondral bone, and saved in the DICOM format, which is standard for storing medical images in PACS. In addition, the range of Hounsfield units to identify bones was 300 to 1300. Then, the DICOM file was analyzed using Analyze 11.0 (AnalyzeDirect, Inc.) for the segmentation of the region of interest (ROI) and transformed into an OBJ file, which was again saved in the STL format using the OBJ Render program (Department of Biomedical Engineering, College of Medicine, Gachon University). Subsequently, the four pieces of the individual 3D models were smoothed using the Meshmixer (Autodesk, Inc.), and each 3D bone model was assembled into a complete proximal humerus after editing it using 3D computer aided design (CAD). We created four 3D bone models with four patients' CT data, but in the last procedure of the finite element model construction, three 3D bone models were inapplicable to the LCP system since the size of humerus head of the remaining three patients was too small and not suitable for attaching LCP. Therefore, we performed the finite element model construction and simulation using data of one bone which was CT data of 80-year-old osteoporotic male patient.

On the other hand, the 3D model for the LCP system (PHILOS, Synthes, Oberdorf, Switzerland) comprising the LCP, locking screws, and cortex screws was built based on the dimensions of real samples (Figure 1(b)) provided by the manufacturer. It is imperative for biomaterials such as a metal implant to meet biocompatibility and thus safety assessments about the exposure to radio frequency (RF) fields must be considered [22, 23]. The LCP system simulated in our work obtained safety-related certification, and other FEA studies [24, 25] analyzing the implanting effectiveness of the same products were commonly carried out under the assumption that biocompatibility issues already were solved, and therefore, we followed the convention. The specifications of the LCP system are presented in Table 1.

The aforementioned process of data preparation is illustrated in Figures 1(a) and 1(b).

### 2.2. Finite Element Model

As stated in the previous section, we considered two types of osteoporotic fracture models: (1) a three-part fracture model composed of the surgical neck of the humerus, greater tubercle, and shaft and (2) a model with an added medial gap fracture (surgical neck of the humerus) at the three-part fractures [24]. The two models were again doubled to four different models with and without a calcar screw. Figure 1(c) describes the main features of the four models; model A and B do not have the medial gap unlike model C and D, and model A and C have a calcar screw whereas model B and D do not [25].

Ten nodes of quadratic tetrahedral elements with three degrees of freedom [12] were used for the discretization of the humerus models and LCP system so that implements the quadratic displacement behavior and achieves more accurate analysis of 3D objects having a complicated or irregular shape such as a humerus fracture [25]. Mesh convergence study was performed and the element sizes of humerus, LCP, and locking screw were 3 mm, 1 mm, and 0.5 mm, respectively.

### 2.3. Material Properties

Materials in finite element models were assumed to be isotropic, homogeneous, and linear elastic. The mechanical properties of all components of both the LCP system and osteoporotic proximal humerus [26] are arranged in Table 2.

### 2.4. Boundary Condition

With regard to the contact conditions at the interface of individual components, it was assumed that the four regions of the humerus, i.e., cortical bone, trabecular bone, alternative cartridge, and subchondral, were completely bonded. Friction coefficients were given to allow finite movement on contact surfaces of the fracture bones and on the contact surface between LCP and cortical bone [27, 28]. In contrast, for the LCP system, there was no relative motion between the interfaces of the screw and surrounding bone and the screw and LCP.

Two types of loads were applied to the head center under the support condition that the end of the humerus shaft is fixed. Two types of external forces were tested. One is axial force of 500 N applied in the vertical direction on the top of the shaft (top of Figure 1(d)) [29], and the other is shear force imposed obliquely with 20° from the head of the greater tubercle (bottom of Figure 1(d)) [29]. The two applied loads intended to emulate the external forces that a proximal fracture site is most likely to experience during daily activities; the first one corresponds to weight bearing by the bone in the standing position, and the second one refers to when rising out of a chair or clutch weight-bearing [29].

## 3. Results

The simulations were performed to investigate the concentration and distribution of stresses occurring in three objects: the maximum shear stresses in the cortical bone, the maximum von-Mises stress in the LCP, and the maximum von-Mises stresses in locking screws. The FEA simulations were performed under with the aforementioned two different external forces and four types of 3D models; consequently, 8 simulations produced 24 resulting values.

The focus of this study was to examine whether a calcar screw can substitute medial cortical support from the perspective of mechanical analysis. Thus, instead of evenly describing all numerical results, we will more concentrate on the stress distribution of the three individual objects in model C against the two applied forces.

The bar graph in Figure 2 compares the simulation results of each model relative to the six categories, and the numerical results are presented in Table 3. As expected, models A and B demonstrated stability under all testing conditions whereas model D revealed that the stress concentration exceeded the ultimate tensile strength (UTS) in all tests. The red dotted lines traversing each bar graph represent the UTS values corresponding to each object.

In terms of the stress concentrations in model C on application of axial forces, a maximum shear stress of 118.5 MPa in the cortical bone appeared in the right side of calcar screw hole as shown in Figure 3(a). In addition, there were a maximum von-Mises stress of 411.32 MPa at the edge of a cortex screw hole on the LCP (see Figure 3(b)), yet the amount of the stress remained within a UTS of 550 MPa. Likewise, the screws under the same simulation showed a maximum von-Mises stress of 351.83 MPa, marked with a red label in Figure 3(c), around the body of the calcar screw, which was significantly lower than a UTS of 900 MPa. To summarize, this model demonstrated that in absence of the cortical medial support, the calcar screw can markedly reduce the stress concentration to a safe level.

Figure 4 displays the results of the shear stress test in model C with respect to the three objects. Cortical bone showed the maximum concentrated shear stress on the edge of the humerus shaft as highlighted with the red label equivalent to 251.10 MPa in Figure 4(a). We will discuss the implication of this result in the next section. As for the stress concentration in the LCP, similar to the analysis with the axial force, a maximum stress of 788.66 MPa developed on the edge of the cortex screw hole but the magnitude of the concentrated force exceeded a UTS of 550 MPa as depicted in Figure 4(b). Although this value indicates a failure from the view of the tolerance limit of the material, the significance of the result must be interpreted based on the extent of deformation and loss of function in the area predicted to be broken. We will discuss this in detail later. Lastly, the calcar screw showed a maximum stress of 663.40 MPa on the head, as shown in Figure 4(c), confirming the successful distribution of the external force within the safe level.

## 4. Discussion

In this work, the effectiveness of the medial screw support for complex fractures at the osteoporotic proximal humerus of the elderly was investigated through computer modeling, focusing on the cases where two routinely encountered external forces were applied to the implanted region. Additionally, we offer visual and quantitative evidence to predict the fixation condition of the LCP in elderly patients, taking advantage of the 3D model virtually realizing real biomechanical structures of the proximal humerus [30] and considering the physical properties of osteoporotic bones. We have also guaranteed the reproducibility of the results by providing the details of the experimental conditions and of the process of reconstructing 3D computer models from raw data and material information of the LCP system. Indeed, to the best of our knowledge, although the mechanical behavior of the medial support in a proximal humerus fracture has been extensively studied through FEA, the effectiveness of the calcar screw for proximal humeral fractures in the elderly with low bone density had not been studied through FEA until now.

The main contribution of this work is twofold. One is the suggestion of four FEA models representing implanting architectures to address the complex fracture of an osteoporotic proximal humerus in elderly patients. The other is the results of the FEA performed to confirm if the calcar screw can substitute medial support in the model with a medial gap.

We obtained 24 resulting values in 8 simulations (Table 3 and Figure 2) revealing the mechanical behaviors of the fixation state with respect to the four models characterized with the presence or absence of medial gap and calcar screw. The results allowed us to observe the distribution and concentration of stresses at specific sites of the virtual specimens and examine both the effect of the calcar screw and the influence of medial support.

More specifically, the fixation approaches for fractured bones in models A and B led to stress distribution within a safe level in view of the ultimate tensile strength (UTS) for both types of external forces; 12 bar graphs corresponding to the maximum stress in models A and B shown in Figure 2 exhibit far less values than the UTS. Considering safety, the LCP and locking screw showed 5.0 and 5.8 of safety factor, respectively, assuring structural safety in both models. In terms of the role of the calcar screw, it was confirmed that, without the medial gap, the contribution of the calcar screw is marginalized (Figures 2(a) and 2(b) and Table 3). In other words, the extent of stress reduction led by calcar screw was insignificant, with an average reduction in stress of <4% in six cases of two forces being applied to the cortical bone, LCP, and screws. Rather, in a few cases in which shear force was applied, introducing calcar screw in model A increased the stress compared to model B, in spite of a negligible level. It would be interesting to examine the cause and effect of this finding because although challenging, it will greatly benefit future FEA studies associated with the medial screw support to uncover the mechanics of the calcar screw in response to external forces and the complexity of the designed model. Based on the stress distribution in models A and B, the combination of the two medial supports does not have any advantage toward reduction of stress concentration.

On the other hand, to evaluate implant-related fixation with respect to the calcar screw when there is a lack of medial support, we compared models C and D; both models lacked medial cortical support, but the former was reinforced with medial screw support as depicted in Figure 1(c). First, the stress concentration in model D immensely exceeded the UTS values in the implant devices and cortical bone, which undoubtedly indicates fixation failure and must be discouraged. In contrast, the adoption of medial screw support dramatically reduced the maximum von-Mises stress of LCP under an axial force of 500 N by 73% from 1550.30 MPa to 411.32 MPa compared to the counterpart without the calcar screw. The contribution to stress distribution was similarly observed by measuring the maximum von-Mises stress in the screw under axial and shear forces, where the maximum stresses were lower than that in model D by 61% and 48%, respectively. Exceptionally, according to the bar graphs of the second group in Figure 2(b), the maximum von-Misses stress loaded on the LCP were greater than the UST value, representing breakage of the device, and this might be interpreted as equivalent to fixation failure. However, it is worth identifying the exact site at which this value was found since qualitative evaluation related to the extent of damage and shape of destruction could supplement the quantitative results. When analyzing the color maps of Figures 3 and 4, aiding visualization of stress distribution and concentration, a maximum stress value of 788.66 MPa appeared on the edge of the LCP cortex screw hole, which indicates local damage affected by a transiently soaring contact pressure at the interface of the screw and LCP. Accordingly, it would be hard to say if the load has enough impact to deteriorate the stability and fixation state of the implant. Based on this comparison, we confirmed that, as far as the absence of medial cortical support is concerned, the calcar screw could be a suitable choice to compensate for the lack of medial support. On the other hand, one may argue that it is not clear whether the benefit was created simply by the increased number of screws. However, previous studies using cadaver have commonly shown that the findings are due to not an increase in the number of screws, but the effect of calcar screws [31].

In conclusion, to secure the stability of the LCP system fixation of a proximal humeral fracture, medial support should be reinforced, and models B and C can be reckoned as complementarily adoptable implant manners depending on the fracture modes related to the medial gap. Even though it is true that model C did not demonstrate stability comparable to medial cortical support, in the case of comminuted fractures, where adequate repair of medial cortical support is challenging, a calcar screw could be the second most desirable option to successfully reduce the stress gradient. These findings are consistent with those of studies investigating the clinical impact of calcar screw with regard to surgical fixation for complex fractures [32, 33].

Also, it would be worth introducing other works having examined the efficacy of calcar screws with respect to various test environments.

In line with our findings, several previous studies [31, 34, 35] have demonstrated that adding calcar screws into locking plate improves fixation stability of three-part varus humeral fractures and reinforces medial support of proximal humeral fractures. Other studies have [36–39] commonly reported that calcar screws could play a crucial role in reducing screw perforation or loss of reduction by providing additional stability when a medial deficiency exists. Specifically, they confirmed that the benefits are resulted in by the improvement of mechanical properties like axial and torsional stiffness in implant system. These studies analyzed and examined the efficacy of calcar screws prior to our work, but they could be viewed as biomechanical studies performed using cadaveric proximal humerus of normal bone rather than FEA study for osteoporotic bone we carried out. On the other hand, there was a similar FEA study [40] to our work that predicted to what extent the failure risk could be reduced when using calcar screws in the fracture of proximal humerus. However, it used low-density bones and attempted to evaluate the effectiveness of the calcar screws in the view of strains applied to around the screws, which are obviously different points from our work. In this work, to enhance analysis accuracy, we introduced some novel strategies associated with experimental conditions. The osteoporotic humerus was divided into four regions, i.e., cortical bone, trabecular bone, articular cartilage, and subchondral bone, and the actual physical properties of osteoporotic humerus corresponding to each component were applied. Subsequently, to allow finite sliding on each interface of fractured bones, relevant friction coefficients were set for the contact surfaces. Related works [27, 28] have demonstrated that imposing a suitable friction condition for the contact areas enables more precise emulation of the actual behavior of the objects.

Additionally, it should be noted that this work has some limitations. First, our experiment was performed using the 3D data of the most desirably-shaped bone selected from 50 patient images to exclude data with shapes to possibly undermine the performance of FEA simulation, and as a result, FEA study was used a single bone. Therefore, considering the statistical generality of the results, it is essential to acquire multiple datasets categorized based on patient sex and age. Second, for the convenience of analysis and reduction of computational cost, our simulation considered a simplified model consisting of only dominant factors, excluding complicated anatomical structures, such as muscles and ligaments that do not significantly affect simulation results. Third, the applied loads in the simulation were designed taking into account the clinical environment and the commonly adopted values in previous studies, but it corresponds to more or less torture testing. In fact, an external force of 500 N estimated to be generated in a person weighing 100 kg is an obviously exaggerated value considering the statistics of the average elderly in South Korea. These issues can be tackled by calibration of experimental conditions based on weight data according to age group or applying various load conditions like torque or a fall on an out-stretched arm. Finally, it is necessary to validate the finite element model by comparing the results of biomechanical studies carried out using cadaveric proximal humerus.

## 5. Conclusion

It was confirmed that the restoration of medial support is imperative for reducing LCP implant-related fixation failure rate, and that the calcar screw is a preferable substitute for medial support in the fracture mode with a medial gap. The stress maps compensated for the limitations of numerical results by helping the visualization of the stress gradient and accurately identifying the sites with maximum concentration of the stress. Simulation conditions and finite element models judiciously constructed reflecting the actual environment and patient statistics can further improve the reliability of the FEA to predict successful reduction of the fractured bone and fixation state of osteoporotic proximal humerus fractures.

## Figures and Tables

**Figure 1:** (a) Overall preprocessing, (b) description of locking compression plate system and proximal humerus, (c) details of four finite element models, and (d) illustration of two types of applied loads.

**Figure 2:** Comparison of maximum stresses with respect to four different fracture models grouped by the individual finite element models. The red dotted lines represent ultimate tensile strength (UTS) of locking compression plate (LCP) and screw: (a) result of finite element analysis under 500 N of axial force and (b) result of finite element analysis under 500 N/20° of shear force.

**Figure 3:** Stress maps of model C under axial force conditions: (a) maximum shear stresses on locking screw–cortical bone interface at cortical head and shaft, (b) maximum von-Mises stresses on the locking compression plate, and (c) maximum von-Mises stresses on locking screw.

**Figure 4:** Stress maps of model C under shear force conditions: (a) maximum shear stresses on locking screw–cortical bone interface at cortical head and shaft, (b) maximum von-Mises stresses on the locking compression plate, and (c) maximum von-Mises stresses on locking screw.

**Table 1:** Details of components consisting of locking compression plate (LCP) system used in this simulation are shown. The second row describes the size and length (*L*) of the used items, and the numbers of the last row correspond to the quantity of used items.

Components	LCP	Locking screw Ø3.5 mm				Cortex screw Ø3.5 mm
	Proximal humeral plate 3.5	L = 25 mm	L = 35 mm	L = 40 mm	L = 40 mm	L = 30 mm
Quantity	1	2	2	4	2 (calcar screw)	1

**Table 2:** Material properties assigned to individual the finite element models. LCP: locking compression plate.

Property	LCP system			Humerus			
	LCP	Locking screw	Cortex screw	Cortical bone	Trabecular bone	Articular cartilage	Subchondral
Material	TiCP	Ti-6Al-7Nb	TiCP	Osteoporotic bone			
Young's modulus (GPa)	103	105	103	12	0.250	0.002	3.5
Poisson's ratio	0.3	0.3	0.3	0.3	0.3	0.3	0.3
Ultimate tensile strength (MPa)	550	900	550	—			

**Table 3:** Comparison of maximum stresses applied to each primary component with respect to fracture models and load conditions. LCP: locking compression plate.

Load condition		Fracture model	Max. shear stress on cortical bone (MPa)	Max. von-Mises stress on LCP (MPa)	Max. von-Mises stress on screw (MPa)
Type	Magnitude				
Axial force	500 N	A	50.80	20.54	42.78
		B	53.96	20.69	42.47
		C	118.5	411.32	351.84
		D	261.92	1550.30	913.20
Shear force	500 N/20°	A	65.05	101.15	155.08
		B	64.77	109.15	143.04
		C	251.10	788.66	663.40
		D	687.86	2926.80	1277.50

## Data Availability

If you require data used in this study, please contact this email: jsmech@gachon.ac.kr
